The article "Gene Expression Analysis Reveals Key Genes and Signalings Associated with the Prognosis of Prostate Cancer" was published in 2021. Journal: Comput Math Methods Med.

# Gene Expression Analysis Reveals Key Genes and Signalings Associated with the Prognosis of Prostate Cancer

**DOI:** 10.1155/2021/9946015

**Published:** 2021-08-28

**Authors:** Hao Shen, Yong-Lian Guo, Guo-Hao Li, Wei Zhao, Ling Zhang

**Affiliations:** ^1^Department of Urology, The Central Hospital of Wuhan, Tongji Medical College, Huazhong University of Science and Technology, Wuhan Hubei Province 430014, China; ^2^Department of Medical Administration, Kuitun Hospital of Yili Kazakh Autonomous Prefecture, Kuitun, Xinjiang Province 833200, China; ^3^Department of Pathology, Wuhan No.1 Hospital, Wuhan, China

## Abstract

It is urgent to identify novel biomarkers for prostate cancer (PCa) prognosis and to understand the mechanisms regulating the tumorigenesis for PCa treatment. In this study, GSE17951 and TCGA were used to identify the differentially expressed genes (DEGs). Our study demonstrated that 1533 genes with increased expression and 2301 genes with decreased expression in PCa. Bioinformatics analysis data indicated that these up-regulated genes had an association with the modulation of mitotic nuclear division, sister chromatid cohesion, cell division, and cell cycle. Additionally, our results revealed downregulated genes took part in modulating extracellular matrix organization, angiogenesis, signal transduction, and Ras signaling pathway. Hub upregulated and downregulated PPI networks were identified by protein-protein interaction (PPI) network analysis and MCODE analysis. Of note, 12 cell cycle regulators, comprising CCNB1, CCNB2, PLK1, TTK, AURKA, CDC20, BUB1, PTTG1, CDC45, CDC25C, CCNA2, and BUB1B, were demonstrated to function crucially in PCa development. By detecting their expression in PCa cell lines, we confirmed that these cell cycle regulator expressions were heightened in PCa cells. GEPIA databases analysis showed that higher expression of these cell cycle regulators was correlated to shorter disease-free survival (DFS) time in PCa samples. Our findings collectively suggested targeting cell cycle pathways may offer novel prognosis and treatment biomarkers for PCa.

## 1. Introduction

Prostate cancer (PCa) ranked second amid the widely occurred carcinoma [1] and its morbidity in China increased largely in recent years [2]. In the past decades, numerous regulators were demonstrated to be associated with PCa development. For example, androgen receptor (AR) displayed importantly in PCa tumorigenesis [3]. Recent studies revealed that mutation of SPOP participated in drug resistance and cross-talked with the AR pathway [4, 5]. Nevertheless, the exact biological mechanism underlying in PCa was still unknown. Besides, lacking special biomarkers for PCa prognosis was another confrontation in PCa treatment. To understand the mechanisms and to seek novel biomarkers are urgently needed in PCa.

The unmanageable cell cycle progression was one of the characteristics of carcinomas [6]. Previous studies have demonstrated the dysregulation of cell cycle regulators had an association with human cancers progression. For instance, increase expression of CDKN3 could induce cell viability and cell cycle in PCa [7]. PSCA was increased in advanced PCa and it could promote cell growth and cell cycle of PCa via activating c-Myc [8]. AURKA functioned crucially in the formation of the mitotic spindle [9]. The PLK1-FOXO1 pathway has been found to be a novel therapeutic marker in advanced PCa [10]. A recent study showed that AURKA expression was induced by androgen and its expression was correlated to a worse biochemical recurrence (BCR) rate [11]. AURKA suppression induces PCa cell line DU145 apoptosis [12]. In addition, CCNA2 was identified as a treatment target of PCa via modulating cell cycle [13]. Investigating the expression patterns and functions of cell cycle regulators could be conducive to uncovering novel biomarkers for PCa.

In our literature, TCGA and GSE17951 were applied to screen the differentially expressed genes (DEGs) in the PCa. The molecular mechanism underlying PCa tumorigenesis and progression was further investigated by protein-protein interaction (PPI) networks. The prognostic value of hub genes was validated by PPI network analysis. Taken together, our literature was conduct to understand the hidden mechanism of PCa at the molecular level.

## 2. Materials and Methods

### 2.1. Microarray Data and Data Preprocessing

In order to identify differentially expressed genes in PCa, we screened public datasets with the GEO database and TCGA database. The database with sample counts >100 was selected for further analysis. Finally, two datasets were used in this study, including GSE17951 and TCGA. The normalization of GSE17951 and TCGA datasets was completed by a robust multiarray average (RMA) method under the R 2.6.2 statistical software with an affy package from BioConductor's affy [14]. Both of them were applied to define the differentially expressed mRNAs. LCM and homogenized tissue datasets were, respectively, applied to obtain the final normalization. Log2-transformed values analyzed by RMA represented relative gene expression level. DEGs were defined as the indicated genes with fold changes (FC) ≥2 and *P* values < 0.05.

Cluster 3.0 with average linkage was used to achieve the hierarchical analysis and visualized via the Java TreeView 1.0.5 software.

### 2.2. PPI Network and Module Analysis

The Cytoscape software was carried out to establish PPI network. The STRING database was used to validate PPI information [15, 16]. The DEGs were mapped to STRING and then were evaluated the interplay between these genes. The comprehensive score >0.4 verified by experiments represented two proteins possessed obvious interaction. Besides, the Cytoscape software [17] version 3.6.0 was conducted to visualize the PPI networks. MCODEtool was performed to screen the PPI network module. *P* < 0.05 indicated a significant statistical difference.

### 2.3. Quantitative Real-Time PCR (qRT-PCR)

Whole RNA was isolated utilizing TransZol Up Plus RNA Kit (TransGen BioTech, China). qRT-PCR was conducted using Talent qPCR PreMix (TIANGEN, China) on a ABI7900 (Thermo Fisher Scientific) system as manual instructed. The primers (forward and reverse) specific for genes were listed below:

CCNB2, 5′-CCGACGGTGTCCAGTGATTT-3′ and 5′-TGTTGTTTTGGTGGGTTGAACT-3′CCNB1, 5′- CATGGTGCACTTTCCTCCTT-3′ and 5′-AGGTAATGTTGTAGAGTTGGTGTCC-3′PLK1,5′-CACAGTGTCAATGCCTCCA-3′ and 5′-TTGCTGACCCAGAAGATGG-3′

TTK, 5′-GTGGAGCAGTACCACTAGAAATG-3 and 5′-CCCAAGTGAACCGGAAAATGA 3′;

CDC20, 5′-GCACAGTTCGCGTTCGAGA-3′ and 5′-CTGGATTTGCCAGGAGTTCGG-3′BUB1, 5′-GGAGAACGCTCTGTCAGCA-3′ and 5′-TCCAAAAACTCTTCAGCATGAG-3′PTTG1, 5′-GCCTCTCATGATCCTTGACG-3 and 5′-GCTTGAAGGAGACTGCAACA-3′

CDC45, 5′-GAAGCGCACACGGTTAGAA-3′ and 5′-GTTCACTCCCAGAGCCACTC-3′BUB1B,5′-CAGTCAGACTCTCAGCATCAAGA-3′ and 5′-CGAGGCAGAAGAACCAGAGA-3′

CDC25C, 5′-TGGGCAAATTTCTTGGTGA-3′ and 5′-AAGATCGAGGCAACGTTTTG-3′CCNA2, 5′-GGTACTGAAGTCCGGGAACC-3′ and 5′-GAAGATCCTTAAGGGGTGCAA-3′AURKA, 5′-CGCCCTGTAGGATACTGCTT-3′ and 5′-CAAATATCCCCGCACTCTG 3′

Actin, 5′-GAGCTACGAGCTGCCTGACG-3′ and 5′-CCTAGAAGCATTTGCGGTGG-3.

Actin was selected as internal reference. All the data was calculated by 2^-*ΔΔ*t^ method.

### 2.4. Statistical Analysis

SPSS16.0 (SPSS, Chicago, Illinois, USA) was applied to analyze the derived data. All representative data were shown as the average value ± standard deviation from three separate experiments in triplicate. Comparisons between groups were analyzed by students' *T*-test or Mann–Whitney *U*-test. The overall survival rate (OS) was evaluated by the Kaplan-Meier method. Cox proportional hazards model and positive stepwise procedure were applied to perform univariate and multivariate survival analysis. Log-rank test was applied to analyze the survival difference. *P* < 0.05 (^∗∗^) means significant difference with a 95% confidence level.

## 3. Results

### 3.1. Screening DEGs in PCa

In this section, two generally used datasets, GSE17951 and TCGA, were applied to screen gene expression and identify the DEGs in PCa. TCGA analysis data illustrated that 3416 increase expression of mRNAs and 4749 decrease expression of mRNAs (Figure 1(a)). Meanwhile, GSE17951 dataset analysis suggested that 3894 upregulated mRNAs and 3981 down-regulated mRNAs (Figure 1(b)). By combining these analyses, our study demonstrated 1533 increase expression of genes and 2301 decrease expression of genes in PCa (Figures 1(c) and 1(d)). The DEGs in PCa were further displayed by Hierarchical clustering analysis.

### 3.2. Bioinformatics Analysis of DEGs in PCa

The unknown functions of these DEGs in PCa were forecasted by bioinformatics analysis. Figures 2(a) and 2(b) indicated that upregulated genes had an association with the modulation of mitotic nuclear division, sister chromatid cohesion, cell division, tRNA aminoacylation for protein translation, translation, Metabolic pathways, N-Glycan biosynthesis, RNA transport, biosynthesis of antibiotics, and cell cycle. Additionally, our results revealed downregulated genes took part in modulating extracellular matrix organization, angiogenesis, signal transduction, heart development, cell adhesion, positive regulation of GTPase activity, axon guidance, regulation of transcription, Focal adhesion, pathways in cancer, Proteoglycans in cancer, and Ras signaling pathway (Figures 2(c) and 2(d)).

### 3.3. Identification of Key Genes in PCa

To identify key genes in PCa, the STRING database was conducted to establish PPI networks. The Cytoscape software was carried out to perform MCODE plug-in analysis. 57 DEGs plus 1451 edges and 56 DEGs with 543 edges were separately demonstrated in the top upregulated and downregulated PPI networks (Figures 3(a) and 3(b)).

Then, the potential roles of these key modules were predicted by the ClueGO plug-in of the Cytoscape software.  Figure 4(a) shown that the upregulated PPI network exhibited an association with the regulation of p53 signaling, Oocyte meiosis, and cell cycle.  Figure 4(b) revealed that the downregulated PPI network was associated with the modulation of the Calcium signaling pathway, and Neuroactive ligand-receptor interaction. The uncontrolled cell cycle progression had been regarded as a characteristic of human cancer. 12 cell cycle regulators were revealed to function crucially in PCa progression, including CCNB1, CCNB2, PLK1, TTK, AURKA, CDC20, BUB1, PTTG1, CDC45, CDC25C, CCNA2, and BUB1B.

### 3.4. Increase Expression of Cell Cycle Regulators Was Shown in PCa Cell Lines

Next, we evaluated cell cycle regulators' expression patterns in normal prostate cell line WPMY-1 and 4 PCa cell lines LNCaP, 22Rv1, PC-3, and DU145. Our data suggested that CCNB2, CCNB1, PLK1, TTK, CDC20, BUB1, PTTG1, CDC45, BUB1B, CDC25C, CCNA2, and AURKA were remarkably upregulated in PCa cell lines relative to that in normal prostate cell line WPMY-1. Interestingly, our data revealed that CCNB1, PLK1, BUB1, and CDC25C were increased up to 10 folds in LNCaP, PC-3, and DU145 cells relative to that in the WPMY-1 cell line (Figure 5).

### 3.5. The Dysregulation of Cell Cycle Regulators Was Correlated to DFS Time in PCa

TCGA dataset was further conducted to assess the association between DFS time of PCa patients and cell cycle regulators expression.  Figure 6 displayed that highly expressed CCNB1, PLK1, CDC20, BUB1, PTTG1, CDC45, BUB1B, CDC25C, CCNA2, and AURKA gave rise to the shorter time of DFS in PCa, suggesting that cell cycle regulators could be regarded as prospective biomarkers for PCa.

## 4. Discussion

In our literature, 1533 genes with increase expression and 2301 genes with decreased expression in PCa were assessed using public datasets. We identified key DEGs in PCa after constructing PPI networks and revealed that the upregulated PPI network had an association with p53 signaling and cell cycle regulation, and the downregulated PPI network was linked to the modulation of the Calcium signaling pathway, and Neuroactive ligand-receptor interaction. Here, we focused on uncovering the expression feature and prognostic significance of cell cycle regulators in PCa. Our data revealed that the cell cycle regulators were obviously upregulated and correlated to a shorter time of DFS in PCa.

Accompanied by the occurrence of high throughput data analysis, several researches revealed some regulators participated in PCa progression. For instance, Ye et al. constructed dysregulated mRNA-, miRNA-, lncRNA-, and TF-mediated regulatory networks in PCa [18]. Fang et al. found that BMP2, PPARG, and PRKAR2B were probable biomarkers for the prognosis of PCa [19]. Here, 1533 genes with increased expression and 2301 genes with decreased expression were identified by GSE17951 and TCGA in PCa. Bioinformatics analysis showed the DEGs in PCa were greatly related with mitotic nuclear division, cell cycle, angiogenesis, signal transduction, cell adhesion, and Ras signaling pathway regulation. Additionally, the identification of key regulators in PCa was also analyzed by PPI networks. Our data arrived at conclusions that the pivotal genes with increase expression took part in p53 signaling and cell cycle modulation, and the primary genes with downregulation participated in the modulation of the Calcium signaling pathway, and Neuroactive ligand-receptor interaction.

The unrestrained cell cycle progression had been regarded as a feature of human cancer. Interestingly, we found multiple cell cycle regulators were up-regulated in PCa, including CCNB1, CCNB2, PLK1, TTK, AURKA, CDC20, BUB1, PTTG1, CDC45, CDC25C, CCNA2, and BUB1B [20–26]. Previous studies had shown that these genes functioned crucially in cell cycle progression and were dysregulated in human cancers. For example, CCNB1 and CCNB2 are the crucial regulators of mitosis initiation and interplayed with CDK1 to further adjust the G2/M phases [27]. CCNB1 and CCNB2 were overexpressed in multiple human cancers. BUB1 and BUB1B were reported to be involved in the process of directing kinetochore localization [28]. The PLK1 functioned importantly in modulating mitotic entry, the G2/M checkpoint, spindle assembly, and chromosome segregation and was a mitotic regulator [29]. TTK is the core spindle assembly checkpoint (SAC) kinase and regulates the recruitment of SAC proteins to unattached kinetochores [30]. Among these regulators, AURKA, BUB1, and PTTG1 were demonstrated to be implicated in PCa development. AURKA and PTTG1 were androgen-responsive genes and crucial for PCa viability and cell cycle.

PSA was the clinical biomarker for PCa prognosis [31]. Nevertheless, due to low specificity, PSA testing was still a problem in clinical practice. A few novel biomarkers, such as PCA3 [32], had also been identified recently. Our study revealed cell cycle regulators, including CCNB1, CCNB2, PLK1, TTK, AURKA, CDC20, BUB1, PTTG1, CDC45, CDC25C, CCNA2, and BUB1B were overexpressed in PCa cell lines and tissues. What is more, highly expressed CCNB1, PLK1, CDC20, BUB1, PTTG1, CDC45, BUB1B, CDC25C, CCNA2, and AURKA were greatly related to the shorter time of DFS in PCa. Our literature implied that these genes could be indicated as newly generated and promising biomarkers for PCa.

## 5. Conclusions

Conclusively, we identified DEGs in PCa were associated with p53 signaling, cell cycle, Calcium signaling pathway, and Neuroactive ligand-receptor interaction. Additionally, we found cell cycle regulators, containing CCNB2, CCNB1, PLK1, TTK, CDC20, BUB1, PTTG1, CDC45, BUB1B, CDC25C, CCNA2, and AURKA, were apparently overexpressed and had a correlation with shorter time of DFS in PCa. These analyses supply innovative clues to uncover cell cycle regulators as potential biomarkers in PCa.

## Figures and Tables

**Figure 1:** The DEGs in PCa. (a) 3416 increase expression of mRNAs and 4749 decrease expression of mRNAs were in TCGA. (b) 3894 increase expression of mRNAs and 3981 decrease expression of mRNAs were in GSE17951 dataset. 1533 increase expression of mRNAs (c) and 2301 decrease expression of mRNAs (d) were both in TCGA and GSE17951 dataset.

**Figure 2:** The bioinformatics analysis of the DEGs in PCa. (a, b) The increased expression of genes was related with the modulation of mitotic nuclear division, sister chromatid cohesion, cell division, tRNA aminoacylation for protein translation, translation, Metabolic pathways, N-Glycan biosynthesis, RNA transport, biosynthesis of antibiotics, and cell cycle. (c, d) The downregulated genes were involved in regulating extracellular matrix organization, angiogenesis, signal transduction, heart development, cell adhesion, positive regulation of GTPase activity, axon guidance, regulation of transcription, Focal adhesion, pathways in cancer, Proteoglycans in cancer, and Ras signaling pathway.

**Figure 3:** The PPI networks of key genes in PCa. (a) The top key up-regulated PPI network comprised 57 DEGs and 1451 edges. (b) The top key down-regulated PPI network comprised 56 DEGs and 543 edges.

**Figure 4:** The potential roles of these key genes in PCa. (a) The upregulated PPI was associated with the regulation of p53 signaling, Oocyte meiosis, and cell cycle. (b) The downregulated PPI was associated with the regulation of the Calcium signaling pathway and Neuroactive ligand-receptor interaction.

**Figure 5:** The cell cycle regulators were upregulated in PCa cell lines and tissues. (a–l) CCNB2 (a), CCNB1 (b), PLK1 (c), TTK (d), CDC20 (e), BUB1 (f), PTTG1 (g), CDC45 (h), BUB1B (i), CDC25C (j), CCNA2 (k), and AURKA (l) were remarkably upregulated in PCa cell lines compared to normal prostate cell line WPMY-1. Significance is defined as *P* < .05 (^∗^*P* < .05; ^∗∗^*P* < .01; ^∗∗∗^*P* < .001).

**Figure 6:** The dysregulation of cell cycle regulators had association with DFS time in PCa. (a–j) The higher expression of CCNB1 (a), PLK1 (b), CDC20 (c), BUB1 (d), PTTG1 (e), CDC45 (f), BUB1B (g), CDC25C (h), CCNA2 (i), and AURKA (j) were significantly linked with shorter DFS time in PCa after TCGA dataset analysis.

## Data Availability

Previously reported lncRNAs data were used to support this study and are available at [doi:10.1158/0008-5472.CAN-10-2585]. These datasets are cited at relevant places within the text as references.
